The article "School-Based Comprehensive Strength Training Interventions to Improve Muscular Fitness and Perceived Physical Competence in Chinese Male Adolescents" was published in 2022. Journal: Biomed Res Int.

# School-Based Comprehensive Strength Training Interventions to Improve Muscular Fitness and Perceived Physical Competence in Chinese Male Adolescents

**DOI:** 10.1155/2022/7464815

**Published:** 2022-09-05

**Authors:** Meiling Zhao, Siling Liu, Xiaowei Han, Zhipeng Li, Baoji Liu, Jianquan Chen, Xiaotian Li

**Affiliations:** ^1^Graduate School, Capital University of Physical Education and Sports, Beijing, China; ^2^College of Sport and Art, Shenzhen Technology University, Shenzhen, China; ^3^Faculty of Education, Beijing Normal University, Beijing, China; ^4^Physical Culture Institute, Guangxi Normal University for Nationalities, Guangxi, China; ^5^Zhichun Branch of Zhongguancun Middle School, Beijing, China; ^6^Yu Yuan Tan High School, Beijing, China; ^7^School of Leisure and Social Sports, Capital University of Physical Education and Sports, Beijing, China

## Abstract

**Purpose:**

This research was to see how effective and feasible school-based comprehensive strength training programs are in improving muscular fitness and perceived physical competence in Chinese male adolescents.

**Methods:**

A total of 123 participants (13.46 ± 0.60 years) were randomized to comprehensive strength training intervention group (CST) (*n* = 62) and the control group (CON) (*n* = 61). The training sessions were performed three times a week for ten weeks in CST. Muscular fitness (i.e., muscular strength, power, and muscular endurance) and perceived physical competence were assessed at initial testing and final testing.

**Results:**

The subjects in the CST significantly improved their mean performance in standing long jump (*p* < 0.05), vertical jump (*p* < 0.05), 1 min push-ups (*p* < 0.05), 1 min sit-ups (*p* < 0.05), handgrip strength (*p* < 0.05), and perceived physical competence (*p* < 0.05) after the intervention. Moreover, the CST were greater in standing long jump (*p* < 0.05), vertical jump (*p* < 0.05), 1 min sit-ups (*p* < 0.05), handgrip strength (*p* < 0.05), and perceived physical competence (*p* < 0.05) compared to the CON, but no in 1 min push-ups (*p* > 0.05).

**Conclusions:**

The comprehensive strength training interventions designed in this study can significantly increase male adolescents' muscular fitness, especially in the lower extremity muscle power and abdominal core endurance, and can enhance their perceived physical competence.

## 1. Introduction

The World Health Organization (WHO) recommends that children and adolescents should engage in a minimum of 60 min of moderate-to-vigorous physical activity (MVPA) every day and at least three days per week of muscle-strengthening exercises (MSE) [1–3]. The health benefits of meeting MVPA and MSE exercises during adolescence are well known such as aerobic fitness[4], muscular fitness[5, 6], skeletal health[4, 7], mental health[8, 9], and metabolic function[10]. However, current data emphasizes the global prevalence of inadequate physical activity among school-aged adolescents, with research indicating that 84.3% of Chinese students (global 81% students) aged 11-17 years were insufficiently physical active in 2016[11]. Furthermore, less than two-fifths of Chinese children and adolescents met the World Health Organization muscle-strengthening exercise recommendations in 2021[12]. Since children and adolescents do not engage regularly in a variety of physical activities, they may be prone to the inevitable consequences of lower muscular fitness and low motor competence.

The term “muscular fitness” refers to three elements of musculoskeletal functioning, namely, maximal strength, muscular power, and local muscular endurance[13]. A growing body of evidence has showed the many benefits of muscular fitness with for a variety of health-related outcomes in adolescents (i.e., body mass index, skinfold thickness, insulin resistance, triglycerides, cardiovascular disease risk score[14], quality of life, attenuate fatigue[15], skeletal health, self-esteem[16], and cognitive task)[17]. Despite the growing number of researches supporting the benefits of muscular fitness, it is often an overlooked element in physical activity guidelines[18]. Many studies have shown a downward continuous trend in muscular fitness among school children in different countries or regions such as the U.S.[19], Britain[20], Canada[21], Spain[22], China[23], and New Zealand[24]. Low muscular strength in teenagers is a developing risk factor for major causes of mortality in early adulthood, such as suicide and cardiovascular diseases[25], and muscular strength in males is inversely and independently associated with death from all causes and cancer[26]. Poor muscular fitness has been linked to pediatric dynapenia in modern-day youth[27] and sarcopenia in elder individuals (i.e., the loss of skeletal muscle mass associated with aging, neuromuscular factors independent of muscle size contribute to muscle weakness, fall risk, declining quality of life, and loss of functional movement)[28, 29]. Furthermore, lower muscle strength was linked to lower cardiorespiratory capacity and motor competence[30, 31]. A number of negative effects of poor muscle strength highlight the need to address the downward continuous trend in muscular fitness among school-aged children.

Perceived physical competence refers to the assessment of adolescents' self-perception in the physical domain[32]. In the physical activity domain, perceived competence is often associated with the confidence in one's ability to take part in sports and outdoor games[33]. Perceived physical competence was positively and substantially connected to physical activity (PA) in males; changes in perceptions may be crucial elements of motivation for PA in school children[34]; it was regarded as a significant factor of behavior[35]. Muscular fitness or cardiorespiratory fitness is associated with motor competence from childhood to early adulthood[36], children with low motor competence demonstrated lower perceived competence[37], and low values in perceived motor competence and actual motor competence and fitness will show a higher probability of maintaining unhealthy lifestyles[38]. Previous studies have looked into the link between motor competence, physical fitness, and perceived motor competence. However, longitudinal intervention studies to increase perceived motor ability are relatively limited. Because boosting male teens' perceived physical competence will be an effective technique for addressing the problem of insufficient physical activity, it is crucial to explore how to improve perceived physical competence.

According to those reviews that summarize the substantial effects of school-based interventions for promoting muscular fitness[18, 39], strength training appears to be one of the most successful PA in teenage boys. Schools are ideally placed to introduce young people to a multitude of lifelong physical activities (including strength training)[40]. However, most school-based PA programs have emphasized aerobic exercises, with relatively few targeting strength training[7]. To find out why, we conducted in-person or phone interviews with 58 secondary school physical education (PE) teachers. Considering the safety of strength training (ST) and the lack of interest of students, they rarely do strength training in PE lessons, despite strength training is safe. Additionally, there is a lack of understanding and knowledge of strength training, and teachers are unclear how to incorporate strength training into regular physical education sessions. Given the importance of muscular fitness for health, there is a need to find a practical and sustainable program. Although recent studies have shown that comprehensive school-based PA interventions are efficiently to improve the cardiorespiratory fitness, muscle strength, and PA[41, 42], the effects of comprehensive school-based strength training interventions on muscular fitness and perceived physical competence of adolescent boys are uncertain. Thus, the purpose of this paper was to determine the impact of comprehensive strength training interventions on muscular fitness of secondary school-aged teenagers (main outcome). The secondary goals were to see if comprehensive strength training interventions affected perceived physical competence. It was hypothesized that after completing the comprehensive strength training interventions program, participants' muscular fitness and perceived physical competence would increase.

## 2. Methods

### 2.1. Participants

The subjects recruited for our study were convenience sample. Participants were required to be healthy adolescents with no history of orthopedic, musculoskeletal, or neurological issues that may have impaired their ability to complete the strength training program and the strength tests. None of the students were athletes, and none of them had ever engaged in organized resistance training. A total of 143 students were recruited for this study. Two were removed because they did not meet the inclusion requirements, leaving 141 healthy boys aged 12-14 years to participate in this study. All eligible students provided written informed permission from their legal guardians. By drawing lots, students were allocated to either comprehensive strength training intervention group (CST) or control group (CON). The CST contained 70 individuals, whereas CON had 71 participants. At any time, any participant might withdraw from the research. Because some students were missing in the posttest or transferred to another school for health reasons, 18 students were omitted from the final analysis after a 10-week intervention. Finally, the effects of the intervention were examined in 123 pupils. At baseline, there were no significant variations in age, body height, body mass, or body mass index (BMI) across groups, as shown in Table 1. The study protocol was approved by the Ethics Committee of Capital University of Physical Education and Sports (code 2022A20), abiding by the Helsinki Declaration amended in Fortaleza (Brazil) in 2013.

### 2.2. Study Protocol

Subjects were recruited from 4 separate physical education classes at the same secondary school. Classes were assigned at random to either a CST or CON. The intervention was founded on the theory of planned behavior[43] and social ecology model[44], and it intended to satisfy students' psychological needs for interpersonal contact, confidence, and intention to engage in school sports and strength training. Before the experimental intervention, PE teachers in the CST were trained to implement the intervention plan. Professional development and equipment (such as resistance bands or dumbbells) were offered to teachers in order to deliver resistance-based exercise. Based on past research, the CST program was particularly designed to be time-efficient, developmentally suitable for teenagers[45, 46]. A graduate student and two PE teachers were on hand to help during the intervention. The CST program included a circuit of 6–8 exercise stations aiming to strengthen muscular fitness (i.e., upper body muscle, low body muscle, and core muscle). Before starting interventions, the subjects in the CST received two weeks of strength training videos, approximately 20 minutes each time, twice weekly, learning by Internet in the classroom to understand the benefits of strength training and master the right skills or methods of RT through power point shows (PPT). After that, a 10-week strength training program was conducted on the playground, with strength training taking place three times a week, on nonconsecutive days, during the first 20-25 minutes of the 45-minute PE class. Participants completed two workouts at each station on the circuit while listening to music, chosen by the adolescents.

According previous studies, youth strength training plans should begin with 1 to 2 sets of 6 to 15 repetitions of each exercise [47]. Starting a strength training program for youths with 10 to 15 repetitions not only brings positive changes in muscular performance but also makes suitable adjustments [6]. In general, when a youngster can comfortably accomplish 15 repetitions, resistance can be raised by 5% to 10% [48]. If the individual fails to finish at least 10 repetitions on each set or maintain appropriate technique[49, 50], the weight is likely too heavy and should be adjusted. It is critical to realize that not all workouts require the same number of sets and repetitions. Thus, participants of this study work in pairs to finish 2 sets of each exercise for 10–12 repetitions in 1-5 weeks (6 exercises including 2–3 resistance band exercises and 3–4 body weight exercises). In weeks 6–10, they did 3 sets of 8–10 repetitions for each exercise using dumbbells (i.e., 0.75 kg, 1.5 kg, and 2 kg) and body weight exercises (for more details, see Table 2). Following a warmup that included dynamic movements or stretching, participants always worked in pairs so that one student was training and the other was observing the partner's performance. Further, all teachers used positive or encouraging phrases to raise the students' perceived of their motor competence. All sessions were recorded and monitored by the authors of this study.

During the 10-week intervention period, participants in the CON went to their regular physical education classes (also three times a week) and were mostly taught volleyball and football. In general, in Chinese regular PE classes, students run for 2-3 laps around the playground before the PE teachers teach them ball skills or other sport programs. During their physical education lessons, no specific resistance exercises were undertaken. Following the study's completion, participants in the CON were provided the strength training courses. All subjects were not allowed to change their daily sports activities during the intervention.

### 2.3. Study Procedure

Within the first minutes of their PE class, the participants in the CST undertook a series of exercises, while the participants in the CON attended their regular PE class as part of the school's curriculum. Data was obtained before and after the intervention. Measurements were chosen to complete a full body muscle strength assessment and to overcome typical challenges to establish a school-based fitness assessment (e.g., lack of resources and insufficient time). Permission to conduct the study was secured from school principals and PE teachers, and participants were informed that their participation was completely voluntary and that they might withdraw at any moment.

### 2.4. Measures

#### 2.4.1. Muscular Fitness

The standing long jump was used to assess the lower body's explosive strength. Participants were asked to stand shoulder-width apart behind a line drawn on the ground and attempt to jump as far as possible they could without falling backwards. A two-foot take-off and landing was used, with forward force produced by swinging of the arms and bending the knees. The distance between the take-off line and the back of the participant's heels was measured. The longest distance was measured to the nearest centimeter after three attempts. The standing long jump is a component of the physical fitness test battery in China, and it is regarded as a valid and reliable field-based assessment of muscular fitness in teenagers[51].

The vertical jump test was used to assess the lower body power. The vertical jump was started at a semisquat position (90° knee flexion), confirmed by eye inspection. Participants held this stance for 2 seconds before jumping vertically for maximal height at the tester's instruction[52]. During the semisquat jump, each participant was carefully examined to ensure that no countermovement was used. Participants lined up at the starting line and leapt as far as they could when the tester signaled. Hands were kept on the hips during the exercise, and participants were advised to keep their lower limbs completely extended throughout the flight. On the portable contact mat, participants were instructed to accomplish 5 consecutive maximum vertical rebounds. Participants were instructed to maximize jump height and minimize ground contact time. All jumps were done on a movable contact mat.

The push-ups were developed to assess upper-body physical endurance[53]. All males were encouraged to do push-ups on their toes, and each student repeated as many push-ups as possible (set at 40 beats per minute), consecutively without rest. The beginning position is in a high plank posture, hands pointing forward and under the shoulder, back straight, head up, using the toes as the crucial point. They had to lower themselves in a controlled way until their elbows formed a 90° angle before returning to the starting position. The test was halted, when the participants strained violently or were unable to maintain the right technique after two repetitions. The maximum number of successfully executed push-ups was recorded, independent of duration.

One-minute sit-up test was used to assess abdominal strength[54]. Participants sat in a supine posture, knees bent at a 90° angle, feet flat on the floor, legs slightly apart, and fingers interlaced behind the head, with a partner holding their ankles firmly to maintain the feet on the ground. The participant's elbows had to contact the knees with an upward movement, and then the two sides of the scapula should return to touch the floor. During 60 seconds, the goal was to repeat this exercise as many times as possible. The test was not counted if the individual failed to contact the knees with his or her elbows, maintain fingers clasped behind the head, or return his or hers to the floor. In 60 seconds, the maximum number of accurately done sit-ups was recorded. Sit-ups, which are also part of the physical fitness test battery in China, are a common way to assess abdominal/core endurance and are safe for children and adolescents to undertake.

A portable handgrip dynamometer was used to test grip strength (CAMRY EH101, China). It is inexpensive and may be utilized in a timely manner. They were instructed to squeeze the dynamometer as hard as they could for 3 seconds after calibrating the dynamometer handle to meet each participant's hand size and their elbow fully extended and adjacent to their torso[53]. All individuals completed three trials of their dominant hand with at least 60 seconds of rest between attempts, and the best performance was recorded. In children and adolescents, handgrip strength has been demonstrated to be associated with muscular strength[55] and has high validity and reliability[56].

#### 2.4.2. Perceived Physical Competence

A French scale was chosen to assess perceived physical competence[57]. It includes endurance, physical strength, and sports competence items, on a 6-point Likert-type scale. A composite score (i.e., average of the four items) was employed for analysis.

### 2.5. Statistical Analysis

The statistical analysis was carried out in IBM SPSS version 24.0. Descriptive data was presented as the mean ± standard deviation (*M* ± *SD*) for all variables. To examine if the changing body mass and height of this rising population will impact any outcome factors, a *t*-test was used to look for group differences in demographic parameters (age, body weight, body height, and BMI) as well as all baseline outcome variables. The interactions and main effects of time (pre- *vs.* posttest) and group (CST *vs.* CON) on the dependent variables were investigated using a repeated measure analysis of variance (ANOVA) (2 × 2). If interactions and main effects were significant, Tukey's LSD post hoc *t*-tests were employed to find specific between-group differences. Partially, eta-squared (*η*_*p*_^2^) effect sizes were estimated within and between groups, and *η*_*p*_^2^ was graded as modest (0.01), medium (0.06), or large (0.14) by Cohen [58]. Statistical significance was set at *p* < 0.05.

## 3. Results

A total of 123 participants finished the 10 weeks strength training program and none of them had a training-related injury. The CST had an 89% attendance at training sessions, whereas the CON had an 86% participation rates in regularly PE class. The demographic factors including age, body weight, body height, and BMI showed no changes between the CST and CON (age: *t*(121) = −0.1, *p* = 0.92; body height: *t*(121) = −1.82, *p* = 0.07; body weight: *t*(121) = −1.18, *p* = 0.24; BMI: *t*(121) = −0.62, *p* = 0.54). Repeated measures variance results showed that the standing long jump (*F*(1, 121) = 28.03, *p* < 0.001, *η*_*p*_^2^ = 0.19), vertical jump (*F*(1, 121) = 37.21, *p* < 0.001, *η*_*p*_^2^ = 0.24), 1 min push-ups (*F*(1, 121) = 17.07, *p* < 0.001, *η*_*p*_^2^ = 0.12), 1 min sit-ups (*F*(1, 121) = 16.02, *p* < 0.001, *η*_*p*_^2^ = 0.12), handgrip strength (*F*(1, 121) = 17.55, *p* < 0.001, *η*_*p*_^2^ = 0.13), and perceived physical competence (*F*(1, 121) = 18.12, *p* < 0.001, *η*_*p*_^2^ = 0.13) had significantly interaction effects.

Regarding the mean within-group changes, CST significantly increased the mean changes of standing long jump (*p* < 0.001), vertical jump (*p* < 0.001), 1 min push-ups (*p* < 0.001), 1 min sit-ups (*p* < 0.001), handgrip strength (*p* < 0.001), and perceived physical competence (*p* < 0.001) from pre- to posttests. However, although each outcome variable in the CON increased, no significant differences were found (*p* > 0.05) (Table 3).

With respect to mean between-group differences, CST significantly increased the mean of standing long jump (*p* < 0.05), vertical jump (*p* < 0.01), 1 min sit-ups (*p* < 0.01), handgrip strength (*p* < 0.05), and perceived physical competence (*p* < 0.001) compared with those in the CON after intervention. But no significant interaction and main effects were found in 1 min push-ups (*p* > 0.05) (Table 3, Figure 1).

## 4. Discussion

The main goal of this study was to see how effective a comprehensive school-based intervention was at enhancing muscular fitness and perceived physical competence among secondary school students. The current study discovered that performing three sessions of comprehensive strength training per week for ten weeks during normal school PE classes was effective in improving muscular fitness and perceived physical competence. No injuries were reported in the CST during the trial.

Muscular fitness is an important aspect of physical fitness. Our findings indicate that a regular school-based comprehensive strength training program can help male adolescents significantly enhance their muscle fitness. The evidence for the effectiveness of a regular RT program in the physical education curriculum for improving muscular fitness in adolescents is increasing[54, 59–61]. Furthermore, a review also showed that strength training can be applied safely and effectively in secondary education[39]. In this study, the CST significantly improved their standing long jump and vertical jump performance in two tests compared with the CON. The standing long jump and the vertical jump field-tests are typically used to evaluate lower body explosive muscular strength in children and adolescents[62]. Previous studies utilizing strength training in secondary school PE lessons have found that the lower body muscle strength improves. In the six-week plyometric training program[59] or in the resistance and combined training groups (plyometric exercises and traditional strength training exercises)[61], horizontal jump distance and vertical jump height increased significantly. Push-ups and sit-ups were used to assess upper-body muscular endurance and abdominal strength. Our study found that the CST increased their sit-up performance in two tests and substantially varied from the CON, but push-ups only found significant improvement in within group effect. The results are partly support by one study[63] which found significant differences between the resistance training group and the control group, when a manual RT program was performance for 20-30 minutes within the PE class, as measured by a pre- to posttest in the push-ups and curl-ups tests. Additionally, a suspension training program twice a week for a total of eight weeks during the physical education class, which included sit-ups and push-ups, resulted in significant variations in baseline values between the intervention group and control group[64]. Another study found that twelve weeks of strength training in PE courses improved push-up and curl-up performance much more than the control group[65]. However, no significant changes in push-ups were seen between the resistance training intervention and control group in another study[66]. The handgrip test is a reliable indicator of upper-body maximum strength in teenagers[51]. The CST improved their handgrip strength in two assessments, and they varied substantially from the CON. This suggestion is in line with the findings of others who have seen substantial improvement in handgrip strength in youth[64, 67]. Contrary to the findings of the present study, no significant gain in handgrip strength was reported following a four-week intervention, when three different programs (aerobic training, RT, and combined training) were compared to a control group [68]. Likewise, after eight weeks of the CrossFit Teens™ resistance training program, there were no changes in handgrip strength in adolescents[69]. This might be related to the fact that the bulk of works with ST equipment requires a strong grip (i.e., resistance bands). Grip strength can also be affected by changes in upper body strength[70]. In addition, we try to understand the significant strength gains from the mechanisms. According to one study, the observed strength gains in youngsters are due to the neural factors rather than muscle hypertrophy[71]. Though training increased muscle strength, intrinsic muscle adaptations (such as changes in excitation or contraction coupling, myofibrillar packing density, and muscle fiber composition) and improvements in motor skill performance and the coordination of the involved muscle groups may also have contributed to the observed strength gains[47]. During and after puberty, adolescents are capable of greater absolute gains owing to higher levels of circulated male hormones [48].

Our findings show that a regular school-based comprehensive strength training program may considerably increase male adolescents' perceived physical competence. This result supports prior findings: higher levels of physical fitness may protect a kid from developing poor motor competence, and low motor competence was associated with lower perceived competence [31, 37]. Adolescence is a critical time for developing lifelong exercise habits, and physical competence appears to be particularly crucial for them. In addition, Jaakkola and colleagues [72] found that moderate-to-vigorous physical activity, perceived physical competence, and health-related fitness (i.e., shuttle run, push-up, and abdominal muscles endurance tests) explained 53% of the variation in motor competence for the boys. Low motor skills, on the other hand, are linked to higher BMI and worse muscle fitness [31]. Many researchers have shown that resistance training may enhance muscular fitness [18, 39, 73]. Therefore, the CST participants' perceived physical competence improved following a brief intervention.

There were several limitations in this study. First of all, due to the teaching arrangement of the school, there was no transit test in this experiment, which meant we could not observe the changes in the experimental group at 5 weeks. In later longitudinal studies, transit testing should be performed if conditions permit. Second, we merely utilized ratings of perceived exertion to determine the intensity of the intervention and did not use objective measures. Finally, there was no follow-up to observe if the changes in muscle fitness (i.e., upper body muscle endurance) and perceived physical competence were sustainable after the intervention.

## 5. Conclusions

It is concluded that the comprehensive strength training interventions designed in this study can significantly increase male adolescents' muscular fitness, especially in the lower extremity muscle power and abdominal core endurance, and can enhance their perceived physical competence.

However, due to the lack of a transit test in this study, we could not obtain valid data on changes in muscle fitness and perceived physical competence at the middle stage of the experiment for male adolescents. Future research should add a transit test to examine the effects of combined interventions. In addition, the exercises of upper body muscle endurance may be insufficient in this programme. It should be paid attention to optimizing the upper body muscle strength training program in future practical application. Finally, considering the importance of muscle strength and perceived physical competence for adolescents, school teachers and policymakers should take effective measures to enhance the muscle strength and perceived physical competence of young people so as to adequately prepare them to participate in higher levels of physical activity.

## Figures and Tables

**Figure 1:** Intervention effects on muscular fitness and perceived physical competence. CST: comprehensive strength training interventions group; CON: control group; ns: no significant group differences; ^∗^*p* < 0.05 difference between CON *vs.* CST; ^∗∗^*p* < 0.01 difference between CON *vs.* CST; ^∗∗∗^*p* < 0.001 difference between CON *vs.* CST.

**Table 1:** Descriptive characteristics of the study participants.

Variables	All (*n* = 123)	CST (*n* = 62)	CON (*n* = 61)
Age (year)	13.46 (0.60)	13.46 (0.55)	13.45 (0.64)
Body height (cm)	165.13 (8.21)	166.45 (7.81)	163.78 (8.45)
Body mass (kg)	58.20 (15.22)	59.79 (14.00)	56.57 (16.32)
BMI (kg/m^2^)	21.23 (4.87)	21.50 (4.45)	20.95 (5.29)

Values are the observed mean (SD); CST: comprehensive strength training group; CON: control group.

**Table 2:** The comprehensive strength training program of the CST.

Week	Content
Week 1	TheraBand–horizontal pull; TheraBand–arm front raises; TheraBand–lunges; TheraBand–squats; single leg hops; sit-ups; partial curls; double crunches
Week 2	TheraBand–horizontal pull; TheraBand–lat pull downs; TheraBand–squats; TheraBand–squat with shoulder press; lateral hops; plank; partial curls; double crunches
Week 3	TheraBand–shoulder lateral raises; TheraBand–lunges with biceps curls; modify push-ups; tuck jumps; jumping lunges; double crunches; double leg raises; plank
Week 4	TheraBand–rowing (sit); TheraBand–shoulder overhead press (sit); TheraBand–calf raises; squats & bicep curls with TheraBand; squat jumps; double leg raises; plank; seated Russian twist
Week 5	TheraBand–triceps kickbacks; TheraBand–lunges with biceps curls; TheraBand–squat with shoulder press; TheraBand–calf raises; tuck jumps; seated Russian twist; double leg raises; plank
Week 6	Dumbbell–biceps curls; dumbbell–reverse fly; dumbbell–squats; dumbbell–lunges; single leg hops; V crunches; reverse curls; plank
Week 7	Dumbbell–lat pull downs; dumbbell–overhead shoulder press; dumbbell–lunges; dumbbell jump squats; jumping lunges; reverse curls; sit-ups with a dumbbell; plank jacks
Week 8	Dumbbell–squat with shoulder press; dumbbell–lunges with biceps curls; dumbbell–split squats; standard push-ups/advanced push-ups; mountain climbers exercise; sit-ups with a dumbbell; plank jacks; advanced Russian twist with a dumbbell
Week 9	Dumbbell–front raises; dumbbell–triceps kickback; dumbbell–lunges with bicep curls; dumbbell–squat with shoulder press; mountain climbers exercise; sit-ups with a dumbbell; leg throw downs; plank jacks
Week 10	Dumbbell–lateral raises; dumbbell–reverse fly; standard push-ups/advanced push-ups; dumbbell–squat with front raises; dumbbell–lateral hops; sit-ups with a dumbbell; leg throw downs; sit-ups

**Table 3:** Effects of the intervention on muscular fitness and perceived physical competence according to group (*n* = 123).

Variables	Pretest *M* ± SD	Posttest *M* ± SD	*Δ* change (95%CI)^a^
*Muscular fitness*			
Standing long jump (cm)			
CST	189.50 ± 3.46	198.34 ± 3.40	8.84^###^ (6.70~10.98)
CON	186.44 ± 3.49	187.15 ± 3.43	0.71 (-1.46~2.87)
*Δ* change (95%CI)^b^	3.06 (-6.68~12.79)	11.19^∗^ (1.63~20.75)	
Vertical jump (cm)			
CST	24.89 ± 5.85	29.70 ± 6.13	4.81^###^ (3.83~5.79)
CON	25.98 ± 6.85	26.52 ± 6.80	0.54 (-0.49~1.52)
*Δ* change (95%CI)^b^	1.09 (-1.19~3.36)	3.18^∗∗^ (0.88~5.50)	
1 min sit-ups (rep)			
CST	39.16 ± 9.52	45.02 ± 9.07	5.86^###^ (4.07~7.64)
CON	39.90 ± 10.10	39.62 ± 10.66	0.72 (-1.08~2.52)
*Δ* change (95%CI)^b^	0.26 (-3.24~3.76)	5.40^∗∗^ (1.86~8.92)	
1 min push-ups (rep)			
CST	20.08 ± 10.02	23.24 ± 10.33	3.16^###^ (2.29~4.03)
CON	20.62 ± 8.35	21.20 ± 7.65	0.57 (-0.31~1.45)
*Δ* change (95%CI)^b^	0.54 (-3.84~2.75)	2.04 (-1.21~5.30)	
Handgrip strength (kg)			
CST	29.65 ± 6.36	31.75 ± 6.83	1.74^###^ (0.99~2.48)
CON	28.02 ± 7.72	27.69 ± 7.30	0.05 (-0.70~0.79)
*Δ* change (95%CI)^b^	1.58 (-0.97~4.12)	3.36^∗^ (0.82~5.90)	
Perceived physical competence			
CST	3.17 ± 0.95	4.05 ± 0.75	0.87^###^ (0.61~1.13)
CON	3.15 ± 1.08	3.23 ± 1.04	0.08 (-0.18~0.34)
*Δ* change (95%CI)^b^	0.02 (-0.34~0.38)	0.81^∗∗∗^ (0.49~1.14)	

CST: comprehensive strength training interventions group; CON: control group; *M* ± SD: means and standard deviation; CI: confidence interval; *Δ* change: mean change prepost treatment; ^a^between-group difference with 95% CI; ^b^within-group difference with 95% CI; ^∗^*p* < 0.05 difference between CON *vs.* CST; ^∗∗^*p* < 0.01 difference between CON *vs.* CST; ^∗∗∗^*p* < 0.001 difference between CON *vs.* CST; ^#^*p* < 0.05 difference between pre- *vs.* posttest; ^##^*p* < 0.01 difference between pre- *vs.* posttest; ^###^*p* < 0.001 difference between pre- *vs.* posttest.

## Data Availability

The data used to support the findings of this study are included within the article. Further information is available from the corresponding authors upon request.
